The article "Effect of Occupation Performance Coaching with Four-Quadrant Model of Facilitated Learning on Children with Specific Learning Disorder" was published in 2022. Journal: Occup Ther Int.

# Effect of Occupation Performance Coaching with Four-Quadrant Model of Facilitated Learning on Children with Specific Learning Disorder

**DOI:** 10.1155/2022/4654204

**Published:** 2022-06-14

**Authors:** Amin Ghaffari, Akram Azad, Mehdi Alizadeh Zarei, Mehdi Rassafiani, Hamid Sharif Nia

**Affiliations:** ^1^Rehabilitation Research Center, Department of Occupational Therapy, School of Rehabilitation Sciences, Iran University of Medical Sciences (IUMS), Tehran, Iran; ^2^School of Allied Health, Exercise and Sports Sciences, Charles Sturt University, Albury, Australia; ^3^Department of Nursing, Amol Faculty of Nursing and Midwifery, Mazandaran University of Medical Sciences, Sari, Iran

## Abstract

**Background:**

Children with a specific learning disability (SLD) have deficits in everyday occupations along with executive function in addition to academic issues.

**Objective:**

The present study is aimed at investigating the effectiveness of Occupational Performance Coaching (OPC) and the Four*-*Quadrant Model of Facilitated Learning (4QM) interventions on the participation in occupational performance and executive function skills in children with SLD.

**Method:**

This study was a single-case experimental design (multiple baselines) in which six children with SLD were randomly assigned to three groups. In the baseline phase, three groups of children underwent repeated executive function assessments using the Stroop Color and Word Test (SCWT) and the Wisconsin Card Sorting Test (WCST) in the multiple baselines. In the intervention phase, all six mothers of children with SLD individually received OPC and 4QM interventions once a week for 14 sessions of 60 minutes and during this period, children were evaluated six more times for executive function skills according to SCWT and WCST. In addition, The Canadian Occupational Performance Measure (COPM) and Behavior Rating Inventory of Executive Function (BRIEF) at the beginning and the end of the baseline phase and the end of the intervention phase were completed by mothers of children with SLD.

**Results:**

More than 50% PND of the SCWT and WCST in the visual analysis graph's information along with significant changes in COPM scores and large effect size of BRIEF subscales (Cohen's *d* ≥ 0.8) in pre- and postintervention showed the effectiveness of OPC and 4QM on the participation in occupational performance and executive function skills in children with SLD.

**Conclusion:**

The results of the study support the effectiveness of OPC and 4QM interventions on children with SLD. However, research with more participants and experimental methods can provide further evidence.

## 1. Introduction

Specific learning disability (SLD) is a neurodevelopmental disorder that is typically diagnosed by low academic achievement and characterized by persistent impairment in reading, writing, and/or math in early school-aged children [1]. The prevalence of SLD in school-age children is reported 5-15% and is two to three times more common in boys than in girls [1]. Even though children with SLD encounter various problems with participation in the activities of daily living, only academic difficulties have received a lot of attention [2–4].

By changing the concept in the diagnosis of learning disability based on DSM-V (Diagnostic and Statistical Manual of Mental Disorders), the focus has shifted from pathology and causality to occupational performance and daily life activities, and the severity of specific learning disabilities is measured according to the child's participation in the occupational performance areas such as self-care (e.g., buttoning up clothes, shoe tying, and climbing up or down the stairs), productivity (e.g., doing homework, legible writing, and organize personal space), and leisure (e.g., painting, playing with peers and reading a book) [1].

Based on the Occupational Therapy Practice Framework (OTPF-4^th^ edition), “participation in occupations is a vital part of human development and life experience, by which it acquires skills and competencies and finds meaning and purpose in life” [5]. In other words, enhancing children's occupational performance which creates a sense of accomplishment and pleasure during childhood helps to encourage positive development into adulthood [6–8]. Therefore, it is important to facilitate the participation of children with SLD in the activities of daily life as the main goal for health professionals and rehabilitation services.

Executive functions refer to a set of cognitive processes, including initiation, planning, decision-making, organization, reasoning, and self-regulation that previous studies in children with SLD have reported defects in executive function skills [9–12]. Children with executive dysfunction may have deficits in managing occupations with dynamic task demands and multiple steps, such as social participation and instrumental activities of daily living, which can lead to restrictions in their life roles [13, 14]. Since executive function skills orchestrate various routine and nonroutine activities of daily living [15–17], therefore, strengthening executive function skills in children with SLD seems necessary to learn new tasks and improve participation in activities of daily living.

According to the International Classification of Functioning, Disability, and Health-Child and Youth (ICF-CY) as a biopsychosocial framework, SLD affect occupational performance and the child's participation in daily life activities [18]. On the other hand, the child's health and well-being are related to the dynamic interaction between body functions/structures (such as executive function skills), activity/participation (such as BADL and IADL) and contextual factors (personal and environmental) [19]. Therefore, by facilitating the child's participation in everyday occupations, in addition to improving executive function skills, the child's independence in occupational performance increases and ultimately reflects better health.

Previous research on children with difficulties shows that the most effective services emphasize the role of the family in treatment [20, 21]. On the other hand, recent qualitative studies on families of children with SLD have stated that improving mothers' learning needs facilitates the teaching of new skills and the solution of problems related to their child's occupational performance [22, 23]. Therefore, empowering mothers of children with SLD, in addition to alleviating the burden and saving time and energy to manage their children compared to their siblings, improves the child's responsibility and participation in daily activities by teaching and learning necessary skills such as executive function skills.

One of the occupation-based, family-centered, and solution-focused interventions is Occupational Performance Coaching (OPC), which empowers mothers to manage their child's barriers to occupational performance by using meaningful and purposeful activities [24]. OPC consists of three main enabling domains including (i) emotional support, (ii) information exchange, and (iii) a structured process [25]. Emotional support involves listening to parents' information and interpretation of the child's occupational performance. During information exchange, a discussion between the mothers and the therapist is done using collaborative performance analysis (CPA) to guide the mother to explore what is currently happening and what they would like to happen and identify bridges and barriers to success and their need to plan and take actions to attain occupational performance goals. In the structured problem-solving process, selected goals related to occupational performance that was chosen by the mother and reflect her concerns for her child begin to explore options between the therapist and the mother. Then, the actions are planned and the results of the actions are checked together [26]. This collaborative approach to problem-solving intends to promote a sense of control and motivate goal achievement using meaningful and purposeful activities [27, 28]. In this way, OPC promotes parental confidence in the ability to teach necessary executive function skills to her or his child, which is important for taking action to overcome barriers in occupational performance [29].

Based on learning theories, systematic facilitator support is needed to teach children new skills to achieve occupational performance goals [30]. In other words, when a child starts the learning process command style (teaching key elements directly to the child along with the way of reacting to task demands) and ends with self-teaching (motivates the child to take into account the challenges to perform the activity through decision-making processes), progress is made toward independence and autonomy in everyday occupation [31]. Thus, selecting effective and systematic teaching-learning strategies seems necessary based on the body functions of children (e.g., executive function skills), mothers' awareness of learning level, and changing needs of children with SLD during the acquisition of new skills to improve taking part in activities daily living.

The Four-Quadrant Model of Facilitated Learning (4QM) is one of the models of learning facilitation in the teaching-learning approach, which was first proposed by occupational therapist Greber et al. [32]. The 4QM provides the various physical and cognitive learning strategies useful in leading children to perform occupational tasks independently [33]. 4QM uses the integration of two continua: (i) directness of the strategy (first direct and then indirect) and (ii) clustering of the initiation source (first, the mother as a facilitator and then the child as a learner) prompt to group learning strategies based on the child's needs. Also, executive function skills such as initiation, proficiency in adaptable thinking, planning, self-monitoring, self-control, termination, time management, and organization, have been used in the quadrants of this model [34]. These strategies are direct and initiated by the mother in quadrant 1. In this quadrant, the characteristics of the task are specified and/or the performance requirements are identified. Other indirect strategies, yet still parent-initiated, fall into quadrant 2 and are useful in encouraging decision-making by the child. Quadrant 3 encourages the child to recall key points through the use of overt self-prompts, and finally, a range of self-regulatory cognitive and metacognitive strategies that are not obvious to observe underpins autonomy in the goals of occupational performance used in quadrant 4 [32].

The OPC approach is potentially effective in improving children's occupational performance by empowering the mothers [28, 29, 35]. On the other hand, with the addition of the 4QM as a reinforcement tool, the OPC can enhance mothers' learning needs and facilitate the teaching necessary skills by mothers to their children with SLD to achieve autonomy and independence in activities of daily life [35, 36].

As far as the authors know, the most recent studies on the participation of children with SLD have examined and identified barriers and facilitators of participation in the everyday occupation of these children [4, 37], and so far, no study has been conducted to facilitate the occupational performance of children with SLD.

Therefore, this study is aimed at investigating the effectiveness of OPC and 4QM interventions on occupational performance and executive function skills as a key prerequisite for goal-directed behaviors and supporting purposeful and meaningful activities in the daily life of children with SLD.

## 2. Methods

### 2.1. Study Design

A multiple baseline single-case experimental design was employed to achieve the selected goals of the current study. This study had two phases including baseline and intervention within which assessment of participation in occupational performance and executive function skills was repeated in both phases.

### 2.2. Participants

Six mothers of children with SLD from special learning problems center No. 1 affiliated to Exceptional Education in Tehran participated in this study. They were randomly divided into three groups. The inclusion criteria for children were (a) ages 7–11 years; (b) diagnosis of SLD by the special learning problems center psychologist approved by the Ministry of Education at the time of registration based on the criteria in the Diagnostic and Statistical Manual of Mental Disorders (5th ed.; DSM–5; APA, 2013); (c) having no visual or hearing problems; (d) having at least an intelligence quotient higher than 70 based on the Persian version of the Wechsler Intelligence Scale for Children Fourth Edition (WISC-IV); and (e) lack of comorbid psychiatric disorder, as measured by the Persian version of Child Symptom Inventory-4 (CSI-4) and referring to the psychiatrist if there were significant symptoms in CSI-4 [38].

In the case of mothers, the inclusion criteria were age between 25 and 50 years and being literate. Mothers were excluded if they were responsible for providing care to another disabled person, had more than one child with a disability, or had severe depression according to the Depression, Anxiety and Stress Scale-21 (DASS-21) [39].

### 2.3. Measurements

The Wechsler Intelligence Scale for Children-Fourth Edition (WISC-IV) was used to measure the intellectual ability of the children in this study [40]. WISC-IV evaluates the combination of verbal comprehension, perceptual reasoning, working memory, and processing speed. The sum of these four subscales provides the overall level of intelligence or Full-Scale Intelligence Quotient (FSIQ). The Persian version of this intelligence scale has acceptable validity and reliability in Iranian students aged 6 to 16 years [41] and can be used to accurately measure children with specific learning disorders [42].

The Canadian Occupational Performance Measure (COPM) was used to determine the therapeutic goals and effectiveness of the intervention on the participation of children in occupational performance [43]. This scale is a semistructured interview that helps mothers to identify goals in the areas of occupational performance (self-care, productivity, and leisure) that their children have difficulty performing. The participating mother was asked to rate her performance and satisfaction with the selected goals related to her child's activities of daily living on a 10-point score (ranging from 1 = not satisfied to 10=satisfied) [44]. Two-point change or more indicates a clinically significant change. Content validity of the Persian version of the COPM was 80.95 ± 0.222 [45].

The Behavior Rating Inventory of Executive Function (BRIEF) was used to assess the behavior and metacognitive function of the child in the natural context, such as home or school [46]. This questionnaire is designed for children aged 5 to 18 years and has been used in a wide range of disorders such as learning disabilities. It consists of 86 items that are divided into 8 separate subscales. The total score of these subscales is named the Global Executive Composite (GEC) which is obtained from the sum of the scores of the two broad scales (behavior regulation index and metacognition index): behavior regulation index (BRI), including inhibition, shifting, and emotional control, and metacognition index (MCI), which includes working memory, initiation, plan/organize organization of materials, and monitoring. The test-retest coefficients in the GEC, BRI, and MCI scales were 0.80, 0.81, and 0.83, respectively [47]. In examining the internal consistency, Cronbach's alpha coefficient for GEC was 0.86 in the Persian version. The Pearson correlation coefficients for GEC, BRI, and MCI were 0.88, 0.83, and 0.84, respectively [48].

The Computerized Stroop Color-Word Test (SCWT) [49] was developed to measure executive function skills such as cognitive flexibility, attention, automation, response inhibition, self-control, and semantic memory. In this neuropsychological test, it takes two seconds to display each stimulus on the computer screen, with a presentation interval of 800 ms between the two stimuli. The stimuli are words with 2 dimensions that include the form of the word and the color of the ink. The answers could be congruent (congruity between the meaning of the word and the color of the ink) or incongruent (differences between the meaning of the word and the color of the ink). The interference score which is considered in this study is calculated as the sum of the Stroop effect (difference between the mean reaction time to incongruent and congruent trials) and Stroop error (difference in the mean number of incongruent and congruent responses). A lower interference score indicates better executive function skills. The Persian version of SCWT software developed by Ravan Tajhiz Sina Company was used in the present study. The internal consistency of reaction times in the three stages was 0.6, 0.83, and 0.97, respectively. Furthermore, internal consistency for error numbers in three stages was also 0.55, 0.78, and 0.79, respectively [50, 51].

The computerized version of the Wisconsin Card Sorting Test (WCST) [52] was used to measure executive function skills such as mental flexibility, abstract behavior, set-shifting, and sustained attention. This test includes images in various shapes (circle, triangle, cross, and/or star-shaped), numbers (1 to 4), and colors (green, blue, red, and/or yellow). Perspective error score was considered in the current study, and a higher score indicates poorer executive function skills. This error is observed when the respondent continues to classify the cards based on the previous principle despite the change of principle by the experimenter or to classify the cards based on a false suspicion and insists on his incorrect answer despite receiving false feedback [53, 54]. This study used version 64 of WCST software developed by Ravan Tajhiz Sina Company. The test-retest reliability of the WCST among the Iranian population was 0.85 [55].

### 2.4. Procedure

According to the inclusion criteria, five boys and one girl were selected from those who were referred to the special learning problems center No. 1 affiliated to Exceptional Education in Tehran. Before entry into the study, all children were tested with the Persian version of the Wechsler Intelligence Scale for Children-Fourth Edition (WISC-IV) to measure their intellectual ability by a special learning problems center psychologist. Then, mothers were interviewed using the COPM to select three goals related to children's participation in occupational performance. Each goal was also rated according to the two sections of satisfaction and performance by the mothers. Furthermore, mothers complete the BRIEF test as an initial assessment.

After completing the outcome measures, six mothers with their children who participated in this study were randomly divided into three groups, and the children were subjected to repeated assessments in two phases including baseline and intervention [56]. In the baseline phase, children underwent repeated executive function assessments using the Stroop Color and Word Test (SCWT) and the Wisconsin Card Sorting Test (WCST). The first group was evaluated for four weeks (12 sessions), the second group for three weeks (9 sessions), and the third group for two weeks (6 sessions), and the results were recorded [57, 58]. In the intervention phase, all mothers individually received Occupation Performance Coaching and the Four-Quadrant Model of Facilitated Learning Interventions. During this period, they were tested six times for executive function according to SCWT and WCST. At the end of the intervention period, mothers score the performance and satisfaction of selected goals in COPM. In addition, mothers complete the BRIEF test as a secondary assessment to evaluate the effectiveness of the intervention, and the results were recorded.

### 2.5. OPC and 4QM Program

OPC and 4QM interventions based on the original OPC protocols [24, 59] consisted of a total of fourteen 60-minute sessions (10 sessions for OPC and 4 sessions for 4QM), which were provided once a week with the first author, who had ten years of experience in pediatric clinical works.

First, necessary explanations about the effectiveness and importance of OPC and 4QM interventions for participation in occupational performance in SLD children were given to the mothers. To make sure of the adherence and compliance to treatment, the evaluation form of the mothers about their ability to implement the programs of each session and the important issues and suggestions during the implementation was completed. Mothers were not required to leave other interventions such as psychology or their child's school tutorials; however, they should have avoided engaging in other occupational therapy interventions.

All participating mothers received a booklet (including printed forms of OPC and 4QM) designed for this study based on previous experience, with information on OPC and additional suggestions on how to implement the 4QM approach along with OPC and guided discovery to support children's participation in occupational performance.

In the first and second sessions, the details of the interventions were introduced separately and in combination with each other, and the mothers were reminded of the three goals related to the children's occupational performance selected by each mother. In the third and fourth sessions, the problem-solving process began for the first goal by completing the booklet of the OPC (problem-solving process) and 4QM (teaching-learning strategies based on the four-quadrant format) given to the mothers. In this session, the mother was asked to carry out two different actions at least along with teaching-learning strategies of 4QM about the desired goal during the next session. In the fifth and sixth sessions, the first goal was reviewed and the problem-solving process on the second and third goals (one or two for each goal) began. After analyzing each goal using collaborative performance analysis in the OPC approach, 4QM was used for the plan action of that goal. In the seventh to twelfth sessions, progress was reviewed across the three goals. In the thirteenth and fourteenth sessions, the selected goals were reviewed and the necessary points for the end of the intervention sessions were discussed.

*OPC approach protocol*. The content of 10 sessions of OPC was based on the enabling principles including three domains: emotional support, information exchange, and structure the process.

In the emotional support domain, listening to parents' information and interpretation of the child was performed. Key facilitating actions in this domain were motivators for change, learning needs in implementing change, and previous success in enabling performance, expressing empathy, assisting parents in reframing their perceptions of the child, enabling performance and guiding parents' reflections and choices of action, and encouraging persistence and future independent problem-solving. In the information exchange domain, discussion took place between the parents and the therapist regarding (a) collaborative performance analysis, (b) understanding typical development, (c) impairments and related challenges in children with SLD, (d) teaching and learning strategies, (e) finding and accessing community resources, and (f) implementation of guided discovery in different settings. Goal setting was done by considering exploring available options in the child (motivation, knowledge, and ability), task (steps of task, sequence of steps, and standard expected), and environment (physical and social) sections.

In this part, by discovering the barriers to accomplishing each goal independently and client-centered in the child, environment, and task sections, essential and required executive function skills in the child section were taught by integrating with the task and environment sections to support their children's participation in occupational performance. Also, action planning, figuring out how to carry out the plan, and checking performance and generalization in the structure the process domain were done [25, 27, 28].

*4QM protocol*. Four sessions of teaching-learning strategies based on 4QM were set in four quadrants during the OPC sessions to achieve the goals that were identified.

In quadrant 1 (task specification), the characteristics and requirements of the task are identified. Strategies are initiated by the facilitator (mother) directly and included explicit instruction/explanation (such as when a mother says to her child: “push your arm through the sleeve”), demonstration (occurs when the mother shows the child how to perform the task), physical patterning (manipulate the child through the entire movement), and lower-order questions (e.g., “what do you do next?”). Attention control and working memory are executive function skills in this quadrant. In quadrant 2 (decision-making), the learner (child) was supported in task performance by encouraging him or her to engage in decision-making processes. Indirect strategies are initiated by the facilitator (mother) and included higher-order questions (e.g., “what might be the problem here?”), feedback (e.g., “Uh-oh, I think there's a problem”), physical prompts (intermittent strategies to ensure motor accuracy using tactile and kinesthetic prompts), nonverbal prompts (e.g., a mother might direct eye gaze at key objects involved in task), and think-aloud modeling (e.g., a mother might comment: “That doesn't seem right. What went wrong there? Maybe if I concentrate on keeping my hand a bit steadier.”). Problem-solving, judgment, reasoning, and decision-making are executive function skills in this quadrant. Quadrant 3 (key points) focused on identifying the steps of the activity and learner- (child) driven processes and highlights direct strategies such as priming (when the child verbally rehearses what he or she will say to the taxi driver while getting out of the taxi), mnemonics (such as acronyms, nonsense phrases, and the use of link words), verbal self-instruction (e.g., a child saying to himself or herself: “I hold it like this and tip it in like that”), visual cues (such as picture cues, computer-generated visual prompts, or mind maps), and kinesthetic self-prompting (strategies enhance the child's attention to a specific action or body part during acquisition skill) that a learner might overtly use to enable his or her performance by focusing on key points. In addition, executive function skills in this quadrant include planning and organizing. Quadrant 4 (autonomy) represents autonomous performance by the learner (child) through indirect strategies such as mental imagery (closing eyes and visualizing doing the task), self-instruction (the use of inner speech to direct the child's actions), self-questioning (the use of inner speech to direct the child's actions), self-monitoring (critiques performance and assesses the need for modification), problem-solving (includes different cognitive processes that are employed to plan, judge, and reason), and automaticity (spontaneous ability to perform a task autonomously). Also, executive function skills in this quadrant include adaptable thinking, self-monitoring, and self-control [32–34, 60].

### 2.6. Data Analysis

The effectiveness of the interventions was determined based on the change in the performance and the satisfaction scores of the children with COPM. A change in score of 2 or more in COPM results indicates a clinically significant change [61].

One of the best methods for data analysis in a single case study is the visual analysis of graph information. For this purpose, first, the data obtained from repeated assessments of executive function skills (SCWT and WCST) in two phases of baseline and intervention were plotted on a graph. In the next step, a line was drawn that exceeds the maximum amount of data in the baseline period and extends in the intervention period. Then, using the statistics of nonoverlap data, it shows the changes in the different phases of the study. Interpretation of the effectiveness of the treatment was performed based on the Percentage of Nonoverlapping Data (PND) according to the following instruction: more than 90% PND means the treatment was very effective; if PND is between 70% and 90%, it means the treatment was effective; if PND is between 50% and 70%, there is ambiguity in the effectiveness of treatment; and PND is less than 50% means that the treatment was ineffective [56].

Also, in order to investigate the effectiveness of the interventions on BRIEF test subscales (BRI, MI, and GEC), the percentage of changes was used in the intervals between the beginning of the baseline phase (baseline A) with the end of the baseline phase (baseline B) and the end of the baseline phase (baseline B) with the end of the intervention phase. Also, the effect size was obtained using Cohen's *d* effect through R software, version 3.5.0. This parameter is calculated as the difference of the means of two phases (baseline A and B+baseline B and intervention) divided by the weighted pooled standard deviations of these phases, and Cohen's *d* = 0.2-0.3, 0.5, and ≥0.8 represent small, medium, and large effect sizes, respectively [62].

## 3. Results

### 3.1. Participants

Six mothers with their children who met the inclusion criteria were selected. All six children are school-aged children aged 8 to 10.5 years who have been diagnosed with SLD. Children 1 and 3 in group one, children 2 and 5 in group two, and children 4 and 6 in group three were randomly assigned. The mean intelligence quotient (IQ) of all children according to WISC-IV was 89.16 (SD = 6.64). Detailed characteristics of the participating mothers with their children are presented in Table 1.

### 3.2. Changes in Performance and Satisfaction of Selected Goals

Table 2 shows the selected goals of the mothers of children with SLD in order of importance, as well as the changes in the rating of the children to the chosen goals in the two sections of performance and satisfaction according to COPM.

Since in the COPM, a change of two points or more indicates a clinically significant change [44, 61], all mothers demonstrated a definitive improvement in both performance and satisfaction for six children at the end of the intervention period. While comparing scores in the baseline period, they did not show a significant difference between the beginning of the baseline phase (baseline A) and its end (baseline B).

### 3.3. Changes in Executive Function Skills

*Executive function changes following SCWT*. This study used the interference score as a dependent variable because it informs on the ability of the child to measure mental flexibility, interference, and response inhibition and allows for the analysis of changes in scores. A lower score reflects improved cognitive flexibility and response inhibition. Interference scores in all children in the baseline period changed slightly, and the lines are almost horizontal, indicating stability in the baseline phase before the intervention phase in all children. However, in the intervention phase, the chart shows an upward trend, and the slope and level of the data indicate an improvement in executive functions. PND related to the interference score of SCWT was “effective” (PND = 83.33%) in four of the children (numbers 1, 3, 5, and 6) and “ambiguity in the effectiveness of treatment/medium effectiveness” (PND = 66.67%) in two of the children (numbers 2 and 4). The PND line drawing also confirms the visual analysis of the data (Figure 1).

*Executive function changes following WCST*. Perspective error score measures set maintenance skills and the ability to flexibly modify incorrect strategies and inhibit incorrect responses. The lower scores of this dependent variable indicate better executive function. PND related to perspective error of WCST was “very effective” (PND = 100%) in three of the children (numbers 2, 3, and 4) and “effective” (PND = 83.33%) in the other three children (numbers 1, 5, and 6). According to the PND line, all six children presented with a score of perspective error during the intervention phase, confirming that the decrease in the score of perspective error was statistically significant (Figure 2).

*Executive function changes following BRIEF*. The results of BRIEF which includes the behavioral regulation Index (BRI), metacognition index (MI), and Global Executive Composite (GEC) showed that all children improved their executive function after the intervention program.

Between baseline phases (baselines A and B), Cohen's *d* values in BRI, MI, and GEC subscales were calculated to be 0.27, 0.38, and 0.33, respectively, so the effect size of the two base phases in all BRIEF subscales was small (Cohen's *d* = 0.2-0.3).

After the interventions, Cohen's *d* values in BRI, MI, and GEC subscales between baseline B and intervention phases were calculated to be 1.40, 1.47, and 1.21, respectively, so the effect size of the end of baseline and intervention phases in all BRIEF subscales was large. (Cohen's *d* ≥ 0.8).

In addition, percentage changes in the subscale BRIEF scores of each child in the beginning and end phases of the baseline (baselines A and B) and the end of the intervention phase are given in Table 3.

## 4. Discussion

This study investigated the effects of OPC and 4QM interventions on occupational performance of selected goals and executive function skills for children with SLD. As indicated by mothers' rating in performance and satisfaction based on COPM, all children have shown significant improvement by increasing two or more points on the selected goals. Furthermore, the results of SCWT and WCST showed stability in the baseline phase, before the intervention phase for each child. All children demonstrated a slope in executive function skills during the intervention phase with a tendency toward improvement. Also, percentage changes and Cohen's *d* value in the BRIEF test subscales showed that the effect size changed from a small effect in the baseline period to a large effect at the end of the intervention period.

The results of the performance and satisfaction scores based on COPM are consistent with the studies by Ahmadi Kahjoogh et al. and Jamali et al., which showed the engagement of mothers in the process of problem-solving related to their children's occupational performance based on the OPC approach [26, 63]. In addition to increasing mothers' motivation and learning needs, they play an active role in achieving their children's goals and may be an important part of the effectiveness of interventions. The development of specific skills required for occupational performance in our study was done using 4QM which confirms the study of Sohlberg et al. about the effectiveness of the systematic instruction approach [36]. Furthermore, our results also support Juntorn et al.'s study which indicated that systematic prompts of 4QM were used to improve the ability of mothers to recall information about how to sequence steps needed for their child's goals [35]. Occupational therapists believe that for health and well-being as the core of the ICF-CY, there must be a balance in the occupational performance areas such as self-care, productivity, and leisure [64]. Thus, we think that using measurements that can analyze everyday occupations in detail may be more beneficial for rehabilitation goals. In this sense, COPM, which helps to assess mothers' perceptions of their child with SLD, can be a guide for creating family-centered interventions using OPC as a problem-solving approach and 4QM as a learning facilitator tool.

At the baseline stage, the children's executive function skills on SCWT and WCST did not change significantly (PND was less than 50%), and this indicates that the time variable or learning effect did not affect repeated administration of SCWT and WCST in three different periods of baseline for these children.

Unlike the baseline phase, at the end of the intervention phase, PND related to SCWT (interference score) and WCST (perspective error) was more than 50% which may be an indicator of the effectiveness of OPC and 4QM interventions on the executive function skills. Our results are similar to findings from studies indicating that there is a significant correlation between executive function skills and occupational performance areas [14, 65, 66]. Therefore, using a top-down approach, the child was helped to perform daily life activities independently and improved executive function skills such as cognitive flexibility, attention, response inhibition, automation, semantic memory, and self-control based on the SCWT and WCST components. Occupational therapists may help mothers of children with SLD resolve problems in their child's occupational performance and provide occupation-based interventions to improve executive function skills through engaging them in meaningful and purposeful activities.

The findings of BRIEF as a parent-report instrument suggested that children's executive function skills in everyday life and various activities had a significant improvement after receiving OPC and 4QM interventions through their mothers [46]. The significant changes in executive function skills found by this method indicated that the changes in executive function skills can be generalized and transferred to different life situations. In the light of these statements, the OPC and 4QM interventions used in this study likely had the characteristics of generalization of skill, which can lead to improving mothers' perspectives of their children's executive function skills in everyday situations. In addition, one of the parts of the problem-solving process in OPC is a generalization and the fourth quadrant of the 4QM also includes problem-solving and thinking strategies; therefore, it seems that the child achieves autonomy in one goal by generalization to other contexts. This seems to be in agreement with the findings of Juntorn et al. and Jamali et al. [35, 63].

Finally, participation in everyday activities is an important aspect of the occupational performance of children with SLD. The OPC approach seems to be an efficient approach to be used as a family-centered, occupation-based, and solution-focused intervention to promote participation in everyday activities. Adding 4QM to OPC, in addition to strengthening mothers' awareness of their learning needs and self-efficacy, may help them better understand their child's level of learning and strive to achieve their occupational performance goals. In summary, considering the effects of participation in occupational performance on executive functions, it appears important to know the relationship between everyday occupations and executive function skills, especially when planning occupational therapy interventions.

### 4.1. Limitations and Suggestions

This study was conducted employing a single-case experimental design and has limited generalizations. It is suggested that in future studies, the effectiveness of the OPC and 4QM interventions in larger sample size and using a control group that only received OPC is examined. This would help to increase the level of evidence and, therefore, the level of generalizability of the results to other similar groups and in other settings such as home, school, and community. The conditions of the studied participants should be examined for longer periods after the intervention to understand the level of stability of the results, level of generalization, and transfers of the learned skills to new tasks and other activities of daily living.

## 5. Conclusion

The single-case design study investigated the effects of OPC and 4QM interventions on participation in occupational performance and executive function skills of children with SLD. The results of this study indicated that OPC and 4QM interventions were beneficial to enhancing scores of performance and satisfaction with identified goals by mothers for the participation of their children along with executive function abilities.

## Figures and Tables

**Figure 1:** Scores for the executive function according to SCWT.

**Figure 2:** Scores for the executive function according to WCST.

**Table 1:** Participants' demographic variables at baseline.

Children	Group	Gender	Age (year)	Level of education	Intelligence quotient (full scale)	Mother's age (year)	Mother's education	Mother's job
Child 1	1	Male	8.50	Second	90.00	40.00	Associate	Housewife
Child 2	2	Male	9.50	Third	90.00	44.00	Bachelor	Employee
Child 3	1	Female	10.50	Fourth	90.00	43.00	Bachelor	Housewife
Child 4	3	Male	8	Second	100.00	38.00	Associate	Employee
Child 5	2	Male	8	Second	80.00	41.00	Bachelor	Housewife
Child 6	3	Male	8	Second	85.00	39.00	Associate	Housewife

**Table 2:** List of the three goals of each child and rating of children in performance and satisfaction according to the COPM.

Children	3 selected goals in order of importance	Performance			Satisfaction		
		Baseline A	Baseline B	Intervention	Baseline A	Baseline B	Intervention
Child 1	Cleaning rooms and personal spaces	1	2	10	1	2	10
	Preparing school bag	1	2	10	1	2	10
	Participate in board games	1	2	8	1	2	7
Child 2	Optimal use of TV and mobile	2	3	10	1	2	10
	Do homework	1	3	6	1	3	7
	Cleaning rooms and personal spaces	1	2	10	1	2	10
Child 3	Participate in cultural and artistic activities	1	1	9	2	2	10
	Activity in social institutions	1	2	9	1	3	8
	Attend extracurricular classes	2	4	9	1	3	9
Child 4	Wearing and taking off shoes	1	1	10	2	2	10
	Do homework	1	3	6	1	2	6
	Bathing independently	1	2	10	2	2	10
Child 5	Preparing school bag	2	2	10	2	3	10
	Performing imaginary games	1	3	8	1	2	8
	Participate in board games	2	3	8	2	2	8
Child 6	Select, wear, and take off clothes	2	3	10	1	2	10
	Play with picky toys like Lego	1	2	8	2	3	8
	Do homework	1	2	7	1	2	8

**Table 3:** Executive function changes following BRIEF.

Children	Baseline A (beginning)			Baseline B (end)			Percentage change (%) (baseline A and B)			Cohen's *d* effect size			Intervention			Percentage change (%) (baseline B and intervention)			Cohen's *d* effect size		
	BRI	MI	GEC	BRI	MI	GEC	BRI	MI	GEC	BRI	MI	GEC	BRI	MI	GEC	BRI	MI	GEC	BRI	MI	GEC
Child 1	54.00	97.00	151.00	52.00	93.00	145.00	-3.70	-4.12	-3.97	0.27	0.38	0.33	45.00	83.00	128.00	-13.46	-10.75	-11.72	1.40	1.47	1.21
Child 2	57.00	100.00	157.00	55.00	96.00	151.00	-3.50	-4	-3.82				43.00	76.00	119.00	-21.81	-20.83	-21.19			
Child 3	53.00	94.00	147.00	50.00	89.00	139.00	-5.66	-5.31	-5.44				42.00	75.00	117.00	-16	-15.73	-15.82			
Child 4	75.00	118.00	193.00	72.00	113.00	185.00	-4	-4.23	-4.14				60.00	100.00	160.00	-16.66	-11.50	-13.51			
Child 5	48.00	85.00	133.00	46.00	81.00	127.00	-4.16	-4.70	-4.51				36.00	63.00	99.00	-21.73	-22.22	-22.04			
Child 6	60.00	100.00	160.00	57.00	97.00	154.00	-5	-3	-3.75				50.00	83.00	133.00	-12.28	-14.43	-13.63			

Abbreviations: BRI: behavioral regulation index; MI: metacognition index; GEC: Global Executive Composite.

## Data Availability

All data used to support the results of this study are included in the article.
